RETRACTED

# Influencing Factors on the Use of Tetrahydrobiopterin in Patients with Phenylketonuria

**DOI:** 10.1155/2022/5245200

**Published:** 2022-07-04

**Authors:** Hui Gao

**Affiliations:** Hebei Shijiazhuang Maternal and Child Health Care Hospital, Shijiazhuang, China

## Abstract

**Objective:**

To explore and analyze the influencing factors of tetrahydrobiopterin therapy in patients with phenylketonuria.

**Methods:**

86 children with phenylketonuria (PKU) diagnosed and treated in our hospital from February 2019 to September 2021 were randomly enrolled. All the children underwent coenzyme hydroxybiopterin and urinary pterin spectrum analysis, and the children with deficiency received gene mutation testing.

**Results:**

The results of urine pterin analysis showed that 82 patients had higher urinary N and B contents than the normal reference values, with the N/B slightly higher than the normal B% within the normal range. 4 patients had extremely high urinary N/B and B% <5% and were diagnosed as BH4 deficiency caused by 6-pyruvoyl-tetrahydropterin synthase (PTPS) deficiency, and a combined stress test was performed. The blood Phe level was (720–1200) *μ*mol/L 3 h after Phe loading, and the blood Phe concentration decreased to (120–240) *μ*mol/L 4–6 h after oral administration of 7.5 mg/kg BH4 tablet. After one week of treatment, the blood Phe concentration decreased significantly to 239 ± 173 *μ*mol/L, with a decrease rate of 52.14 ± 25.28%. It shows that the application of tetrahydrobiopterin intervention therapy is effective in patients with PKU. The results of the full-length cDNA analysis of the PTPS gene showed that a total of 4 gene mutations were found. A C ⟶ T substitution occurred at the 259th base, and the 87th proline (Pro) in the coding region was converted to serine (Ser) (P87S). G ⟶ A substitution at base 286 converts aspartic acid (Asp) at position 96 of the coding region to asparagine (Asn) (D96N). A ⟶ G substitution occurs at the 155th base to convert asparagine (Asn) at position 52 of the coding region to serine (Ser) (N52S). G ⟶ C substitution occurs at the 430th base to convert glycine at position 144 (Gly) to arginine (Arg) (G144R). G144R is a new mutation type. The gene mutation types of the 4 patients were P87S/D96N, N52S/G144R, D96N/P87S, and P87S/P87S, all of which were from their parents, which conformed to the law of autosomal recessive inheritance.

**Conclusion:**

PKU is caused by the defect of phenylalanine hydroxylase activity in children, which causes phenylalanine metabolism disorder, and tetrahydrobiopterin intervention therapy can affect the activity of phenylalanine hydroxylase, increase the decline rate of blood Phe, significantly reduce the level of phenylalanine in children, and promote intellectual recovery. The dose of tetrahydrobiopterin should be tailored, with small doses for mild phenotypes and long-term treatment using even smaller doses.

RETRACTED

## 1. Introduction

Phenylketonuria (PKU), a congenital metabolic disease [1], is caused by phenylalanine metabolism disorder resulting from phenylalanine hydroxylase deficiency in the liver due to chromosomal gene mutation, which often leads to central nervous system damage [2, 3]. In 1934, Folling [4] found a large amount of phenylpyruvate in the urine of 2 siblings with neurodevelopmental delay and named the disease “phenylpyruvate urinary intellectual hypoplasia.” Penrose [5] later confirmed that the main contributor to the disease was the excessive levels of phenylalanine (Phe) in the blood, so the disease was named hyperphenylalaninaemia (HPA) and afterwards named PKU. Phe is one of the essential amino acids in the human body and metabolized via the conversion of coenzyme tetrahydrobiopterin (BH4) into tyrosine (Tyr) under the action of Phe hydroxylase (PAH) [6]. In the event of a mutation in the gene encoding PAH, the activity of PAH synthesized by the liver is reduced or absent, or the deficiency of its coenzyme BH4 will lead to the blockage of the normal metabolic pathway of Phe in the body. As a result, substrates and secondary metabolites are accumulated in the body, and the reduction of normal metabolites and the accumulation of abnormal metabolites will trigger a series of PKU diseases characterized by intellectual impairment [7].

PKU is a treatable autosomal recessive inherited metabolic disease and is categorized as per the different etiologies into PKU caused by mutations in the PAH gene resulting in decreased or loss of PAH activity and BH4D deficiency caused by a congenital defect of an enzyme in the synthesis or metabolism pathway of the coenzyme of PAH (BH4) [8, 9]. Due to the toxicity of HPA and its intermediate metabolites on the central nervous system, these two diseases with different etiologies lead to severe neurological damage and intellectual disability in children. In 1999, Kure et al. [10] found a reduced blood Phe concentration after the oral administration of BH4. BH4-responsive PAH deficiency is divided into complete responders and partial responders [11]. The complete responder means that the blood Phe concentration of patients can reach normal levels after BH4 medication, whereas the partial responder fails to reach the normal range. Despite a certain efficacy of the dietary therapy for PKU [12], there exist key issues such as difficulties in long-term adherence and heavy economic burden to be addressed. Issues associated with dietary therapy include (1) poor compliance with treatment due to poor dietary taste, (2) ongoing neurological and psychological problems due to low quality of life despite early intervention, (3) multiple nutrient deficiencies due to dietary restrictions, and (4) the high cost of special foods and nutrients and the financial burden on families. Dietary control during the neonatal and early childhood periods is relatively easy. However, the compliance with the diet deteriorates as the patient gets older until around puberty. This problem is clearly evidenced by the poor control of blood phenylalanine concentrations in this age group. In recent years, many scholars have dedicated to the exploration of alternative treatments, aiming to find more convenient treatment methods. According to recent studies on BH4-responsive PKU, it has been proposed that the administration of physiological doses of BH4 is an alternative to diet therapy for mild PKU and MHP [13, 14]. Therefore, the purpose of the present study is to explore and analyze the influencing factors of tetrahydrobiopterin therapy in patients with PKU. The current clinical work uses drugs that promote the development of brain cell function as the corresponding adjuvant therapy for PKU. It mainly stimulates brain cells and enhances the repair function of brain cells to refresh the brain, nourish the liver and kidney, promote blood circulation and dredge collaterals, resolve phlegm, and remove blood stasis. The difference between the central nervous system and other systems is that neurons, as the basic unit of the nervous system, are extremely difficult to regenerate after damage caused by various factors, and the original neural circuit and other structures cannot be restored after damage. Therefore, the nervous system must rely on some compensatory functions of the nervous system to maintain the normal life activities and functions of the body. The “multidimensional comprehensive intervention method” in traditional Chinese medicine has achieved good results in the treatment of PKU via multiple solutions such as oral decoction, scalp acupuncture, ear acupuncture, and acupoint injection.

RETRACTED

## 2. Participants and Methods

### 2.1. Participants

A total of 86 children with PKU diagnosed and treated in our hospital from February 2019 to September 2021 were randomly included in this study. Most of the children showed mental retardation and jaundice. There were 47 males and 39 females, with an average age of 0–3 (1.23 ± 0.84) years, with 63 cases of mild PKU (blood Phe: 360–1200 *μ*mol/L) and 23 cases of classic PKU (blood Phe ≥ 1200 *μ*mol/L).

### 2.2. Inclusion Criteria

The inclusion criteria were as follows: ① all met the diagnostic criteria for PKU; ② the patients and their families were informed of the contents of the study and signed the consent form voluntarily; ③ this study was approved by the Ethics Committee of Hebei Shijiazhuang Maternal and Child Health Care Hospital, under No. SJZ8-82987.

### 2.3. Exclusion Criteria

The exclusion criteria were as follows: ① the patients had severe organic diseases; ② the patients had severe mental disorders; ③ the patient's family refused to participate in this study.

### 2.4. Methods and Indicators

#### 2.4.1. Phe + BH4 Loading Test

Those with basal blood Phe < 600 *μ*mol/L first underwent a Phe (100 mg/kg) oral loading test, followed by an oral BH4 (20 mg/kg) loading test 3 hours after the administration of Phe. Peripheral blood was collected on a dry filter paper at 1, 2, and 3 hours before and after taking Phe and at 2, 4, 6, 8, and 24 hours after taking BH4, and the concentration of blood Phe was determined by the fluorescence method. A decrease in blood Phe concentration of more than 30% compared to predose within 24 hours after taking BH4 can be diagnosed as BH4-responsive PAH deficiency after excluding BH4 deficiency.

#### 2.4.2. Urinary Pterin Spectrum Analysis

Urine neopterin (N), biopterin (B) content, and biopterin B% (B/(B + N)) were determined by high-performance liquid chromatography (HPLC) to screen for BH4 deficiency. A deficiency of 6-pyruvoyl-tetrahydropterin synthase (PTPS) in the BH4 synthesis pathway was considered. There was a significant increase in N, a significant decrease in B in the urine, an abnormal increase in N/B, and a B% less than 10%. If there was a decrease in N/B and an abnormal increase in B% in the urine, further determination of dihydrobiopterin reductase (DHPR) activity is required to confirm the diagnosis of DHPR deficiency.

#### 2.4.3. Treatment

With the consent of the patient's family members, 10–15 mg/(kg*∗*d) of BH4 was given on the basis of ordinary diet and the blood Phe concentration was measured.

#### 2.4.4. PAH Gene Detection

Genomic DNA was extracted from peripheral blood leukocytes, and exons of PAH gene were amplified by PCR. The PCR products were screened for mutation by denaturing gradient gel electrophoresis (DGGE), and the abnormal bands were directly sequenced.

#### 2.4.5. Multidimensional Comprehensive Intervention Method

Taking acupuncture points on the head “Four Shen Needles,” “Zhi Three Needles,” “Nao Three Needles,” and “Temporal Three Needles” as the main points, TCM syndrome differentiation and treatment were combined and a period of four months was taken as a course of treatment. In addition, tonifying Qi and essence soup was supplemented for clearing heat and dampness, strengthening the spleen, and draining turbidity: 20 g each of *Coix lacryma* and *Poria*, 18 g of *Astragalus*, 14 g of Rhizoma Dioscorea, 9 g each of *Plantago ovata* and Rhizoma Polygonati, 7 g each of *Pueraria lobata* and *Acorus calamus*, 5 g of Rhei Radix et Rhizoma, and 3 g of *Coix* Seed (1 time a day and 1 month as a course of treatment).

RETRACTED

## 3. Results

### 3.1. Phe + BH4 Stress Test and Urinary Pterin Spectrum Analysis

The results of urine pterin analysis showed that 82 patients had higher urinary N and B contents than the normal reference values, with the N/B slightly higher than the normal B% within the normal range. 4 patients had extremely high urinary N/B and B% <5% and were all diagnosed as BH4 deficiency caused by PTPS deficiency, and a combined stress test was performed. The blood Phe level was (720–1200) *μ*mol/L 3 h after Phe loading, and the blood Phe concentration decreased to (120–240) *μ*mol/L 4–6 h after oral administration of 7.5 mg/kg BH4 tablet, which was further confirmed as BH4 deficiency (Table 1).

### 3.2. Posttreatment

After one week of treatment, the blood Phe concentration decreased significantly to 239 ± 173 *μ*mol/L and the decrease rate was 52.14 ± 25.28%. It shows that the application of tetrahydrobiopterin intervention therapy is effective in patients with PKU.

### 3.3. Genetic Testing

The results of the full-length cDNA analysis of the PTPS gene showed that a total of 4 gene mutations were found. A C ⟶ T substitution occurred at the 259th base, and the 87th proline (Pro) in the coding region was converted to serine (Ser) (P87S). G ⟶ A substitution at base 286 converts aspartic acid (Asp) at position 96 of the coding region to asparagine (Asn) (D96N). A ⟶ G substitution occurs at the 155th base to convert asparagine (Asn) at position 52 of the coding region to serine (Ser) (N52S). G ⟶ C substitution occurs at the 430th base to convert glycine at position 144 (Gly) to arginine (Arg) (G144R), and G144R is a new mutation type. The gene mutation types of the 4 patients were P87S/D96N, N52S/G144R, D96N/P87S, and P87S/P87S, all of which were from their parents, which conformed to the law of autosomal recessive inheritance.

### 3.4. Long-Term Follow-Up

Long-term follow-up of patients after treatment showed that the effect of marrow treatment is promising, but there is still the problem of delayed language development. After research and analysis, the following experiences have been concluded: (1) children who receive treatment within 3 months after birth have significant curative effect and can avoid severe intellectual disability; (2) according to clinical symptoms, specific conditions of patients, and levels of neurotransmitter metabolites in the cerebrospinal fluid, the drug dose should be adjusted flexibly; (3) the blood Phe concentration of precursor should be strictly controlled at <240 *μ*mol/L to avoid the increase of blood Phe concentration interfering with the therapeutic effect.

RETRACTED

## 4. Discussion

PKU is an autosomal recessive metabolic disease caused by a chromosomal gene mutation that leads to a defect in phenylalanine hydroxylase in the liver, resulting in a disorder of phenylalanine metabolism [15, 16]. The lack of synthetase or reductase in the BH4 anabolic pathway reduces the stability of phenylalanine hydroxylase and increases blood Phe [17, 18]. In partial or mild BH4 deficiency, the BH4 produced by the remaining enzymatic activity can still meet the synthesis of neurotransmitters in the brain, manifesting only as increased blood Phe without other neurological symptoms. The clinical treatment of PKU is dietary therapy [19], which features a well-recognized efficacy. However, patients receiving dietary therapy usually experience low treatment compliance and a heavy economic burden, which may be predisposed to recurrence. In recent years, various alternative treatments have been investigated to optimize the treatment methods. Previous research has shown [20] that urine pterin analysis is a commonly used screening method for BH4 deficiency, and BH4 stress test is a more reliable and rapid differential diagnosis method. The results of this study showed that 82 patients had higher urinary N and B contents than the normal reference values, with the N/B slightly higher than the normal B% within the normal range, and 4 patients had extremely high urinary N/B and B% <5%. Therefore, they were all diagnosed as BH4 deficiency caused by PTPS deficiency, and a combined stress test was performed: 3 h after Phe loading, the blood Phe was (720–1200) *μ*mol/L, and the blood Phe concentration decreased to (120–240) *μ*mol/L 4–6 h after oral administration of BH4 tablets of 7.5 mg/kg. This was further confirmed as BH4 deficiency. According to the recent studies on BH4-responsive PKU, it has been proposed that the administration of physiological doses of BH4 (10–15 mg/(kg*∗*d)) is an alternative therapy for the dietary treatment of light PKU and MHP. The results showed that after 1 week of treatment, the blood Phe concentration decreased significantly, and the results showed that the amount of specific decrease was 239 ± 173 *μ*mol/L and the decrease rate was 52.14 ± 25.28%. It is suggested that the application of tetrahydrobiopterin intervention therapy is effective in patients with phenylketonuria. After administration of exogenous BH4, the activity of PAH can be restored to normal and the concentration of blood Phe can be completely reduced to normal 2–6 h after administration of BH4. In 1992, Thony et al. cloned the cDNA of human hepatocyte PTPS, and its gene was located in the 6th exon of chromosome 11 (11p22.3).

RETRACTED

To date, 7 types of gene mutations have been found in Chinese PTPS-deficient patients, among which P87S and N52S are the most common, accounting for 70% and more common in northern and southern China; N52S is more frequently seen in southern patients. The full-length cDNA analysis of the PTPS gene showed that a total of 4 gene mutations were found: a C ⟶ T substitution occurred at the 259th base, and the 87th proline (Pro) in the coding region was converted to serine (Ser) (P87S); G ⟶ A substitution at base 286 converts aspartic acid (Asp) at position 96 of the coding region to asparagine (Asn) (D96N); A ⟶ G substitution occurs at the 155th base to convert asparagine (Asn) at position 52 of the coding region to serine (Ser) (N52S); G ⟶ C substitution occurs at the 430th base to convert glycine at position 144 (Gly) to arginine (Arg) (G144R). G144R is a new mutation type. The gene mutation types of the 4 patients were P87S/D96N, N52S/G144R, D96N/P87S, and P87S/P87S, all were from their parents, in line with the law of autosomal recessive inheritance, and the type of gene mutation was consistent with the clinical phenotype. After research and analysis, the following experiences have been concluded: (1) children who receive treatment within 3 months after birth have significant curative effect and can avoid severe intellectual disability; (2) according to clinical symptoms, specific conditions of patients, and levels of neurotransmitter metabolites in cerebrospinal fluid, the drug dose should be adjusted flexibly; (3) the blood Phe concentration of precursor should be strictly control at <240 *μ*mol/L to avoid the increase of blood Phe concentration to interfere with the therapeutic effect.

Phenylalanine, tyrosine, tryptophan, and some branched-chain amino acids are called macronutrient amino acids, and they cross the blood-brain barrier through a common transport carrier. Therefore, increased phenylalanine concentrations in the blood compete with other large neutral amino acids to cross the blood-brain barrier, and supplementation with large neutral amino acids has been shown to reduce phenylalanine concentrations in the brain [10].

Glycopeptide is a natural low-phenylalanine protein extracted from whey and is rich in valine, isoleucine, and threonine. After purification, glycopeptides mixed with other essential amino acids (tyrosine, tryptophan, arginine, cysteine, and histidine) can be used as a low-phenylalanine diet [6–8]. Dietary formulations containing glyco-macropeptides are better tasting and more acceptable than conventional low-phenylalanine diets. Research has demonstrated that glycopeptide diets significantly reduce urea production and increase phenylalanine utilization [9].

RETRACTED

The recombinant adeno-associated virus (rAAV) in gene therapy for phenylalanine ketonuria is more advantageous as a safer gene introduction vector, as rAAV carries no viral genes and hence elicits a small immune response. It has been demonstrated that rAAV vectors containing mouse PAH cDNA can reduce blood phenylalanine levels after portal vein injection into the liver [19]. However, phenylalanine was again elevated to pretreatment levels after 40 weeks of application of this approach. This is because most vectors are genotoxic through mitosis and can impair the stability of the transferred genes. Thus, further studies are required before the clinical application of gene therapy.

Multidimensional comprehensive intervention in the treatment of PKU is the crystallization of clinical wisdom. It has the effects of adjusting the brain and fu organs and Qi, nourishing the brain and strengthening the brain, nourishing the liver and kidney, filling the essence, nourishing the heart and spleen, promoting the brain development of PKU patients, enhancing intelligence, and improving adaptive behavior disorders. Although there is no record of phenylketonuria in the Chinese medical literature, there are records similar to this disease according to its clinical symptoms. In the Zuo Zhuan, it is described as “unwise, the so-called idiot” or in “The Secret Tale of the Doctor,” it is named as “Dementia.” In congenital dementia, traditional Chinese medicine mainly focuses on tonifying the heart and kidneys, filling the essence, and nourishing the marrow, together with benefiting the Qi and nourishing the blood, correcting the origin, eliminating stasis, and resolving turbidity. The prescription of Chinese medicine contains 20 g each of *Coix lacryma* and *Poria*, 18 g of *Astragalus*, 14 g of Rhizoma Dioscorea, 9 g each of *Plantago ovata* and Rhizoma Polygonati, 7 g each of *Pueraria lobata* and *Acorus calamus*, 5 g of Rhei Radix et Rhizoma, and 3 g of *Coix* Seed, with the aim of clearing heat and dampness, strengthening the spleen, and draining turbidity. In this formula, *Astragalus* and *Poria* tonify Qi and resolve turbidity, Rhizoma Dioscorea, Rhei Radix et Rhizoma, and *Coix* Seed resolve heat and dampness, and Rhei Radix et Rhizoma has the effect of detoxification similar to sodium bicarbonate. The remaining drugs tonify the kidney, promote cerebral circulation, and strengthen the spleen [16]. Acupuncture improves IQ and the expression levels of trace elements in patients with PKU. Studies have shown that trace elements such as Zn (zinc), Cu (copper), Fe (iron), and Cd (cadmium) have a nonnegligible effect on the development of the nervous system in children. The occurrence of PKU is also closely related to the abnormality of these elements [17]. The study showed that the content of Zn, Cu, and Fe in PKU patients increased significantly after acupuncture treatment, while the content of Cd decreased significantly. PKU patients have abnormal trace elements in the body, and acupuncture treatment can adjust and normalize the abnormal trace elements in the body. The normal coordination of trace elements plays an important role in promoting the synthesis of RNA and protein in the brain tissue, in the normal conduction of axonal nerves in the brain tissue such as hippocampus, and in enhancing SOD activity. Multidimensional comprehensive intervention in the treatment of PKU has a positive clinical effect, and it has unique advantages in reducing lipid peroxidation damage in the brain tissue and promoting the synthesis of RNA and protein in the brain tissue, thereby promoting the improvement of clinical symptoms and the recovery of intellectual function.

RETRACTED

## 5. Conclusion

PKU is caused by the defect of phenylalanine hydroxylase activity in children, which causes phenylalanine metabolism disorder, and tetrahydrobiopterin intervention therapy can affect the activity of phenylalanine hydroxylase, increase the decline rate of blood Phe, significantly reduce the level of phenylalanine in children, and promote intellectual recovery in children. The dose of tetrahydrobiopterin should be tailored with mild phenotypes using small doses and long-term treatment using even smaller doses.

## Figures and Tables

**Table 1:** Urine pterin analysis results of all patients.

	Age (year)	Phe (*μ*mol/L)	Neopterin (mmol/molCr)	Biopterin (mmol/monCr)	N/B	B%
PKU	1.23 ± 0.84	961 ± 341	3.63 ± 3.60	5.57 ± 6.01	1.05 ± 1.32	57.92 ± 17.61
PTPSD 1	1.41	360	4.35	0.0100	265.00	0.25
PTPSD 2	0.98	1200	0.019	0.0034	56.30	0.08
PTPSD 3	1.37	360	4.28	0.0101	428.00	0.21
PTPSD 4	2.03	900	1.003	0.0060	165.21	0.31
Reference value	2 months to 6 years	＜120	0.28–2.60	0.35–2.96	0.30–0.94	42.70–75.90

## Data Availability

The datasets used during the present study are available from the author upon reasonable request.
